This article has been retracted.

# lncRNA H19 Aggravates Brain Injury in Rats following Experimental Intracerebral Hemorrhage via NF-*κ*B Pathway

**DOI:** 10.1155/2022/3017312

**Published:** 2022-01-15

**Authors:** Shuaidong Mao, Huan Huang, Xianzheng Chen

**Affiliations:** ^1^Department of Neurosurgery, Shanghai Tenth People's Hospital Chongming Branch, Shanghai 202157, China; ^2^Department of Neurosurgery, Shanghai Tenth People's Hospital, Shanghai 200072, China

## Abstract

**Objective:**

To explore the effect of long noncoding RNA H19 (lncRNA H19) on brain injury in rats following experimental intracerebral hemorrhage (ICH).

**Methods:**

Rat ICH model was established with type IV collagenase. The neurological function scores were evaluated, and the water content in brain tissue was measured. The nerve injury indexes, inflammatory factors, and oxidative stress indexes were also measured. Moreover, the expression of lncRNA H19 was determined by qRT-PCR, and Western blot detected NF-*κ*B pathway-related protein expression.

**Results:**

Compared with the sham group, the neurological function scores, the water content in brain tissue, and levels of injury indicators myelin basic protein (MBP), S-100B, and neuron-specific enolase (NSE) in the ICH rats were significantly increased. Meanwhile, the levels of TNF-*α*, IL-6, IL-1*β*, ROS, and MDA were significantly increased, but the levels of SOD were significantly decreased. In addition, the expression of lncRNA H19 in the brain tissue in the ICH group was significantly higher than that in the sham group. After further interference with lncRNA H19 expression (sh-H19 group), the levels of all the above indicators were reversed and the neurological damage was improved. Western blot results showed that the expression of NF-*κ*Bp65 and IKK*β* was significantly higher, and I*κ*B*α* expression was lower in the perivascular hematoma tissue in the ICH group compared with the sham group. Compared with the sh-NC group, NF-*κ*Bp65 and IKK*β* expression were significantly lower and I*κ*B*α* was significantly higher in the sh-H19 group.

**Conclusion:**

lncRNA H19 exacerbated brain injury in rats with ICH by promoting neurological impairment, brain edema, and releasing inflammatory responses and oxidative stress. This may be related to the activation of NF-*κ*B signaling pathway.

## 1. Introduction

Intracerebral hemorrhage (ICH) refers to primary cerebral intracephalic bleeding, which accounts for 10%-20% of all strokes [1], and is one of them with few effective therapeutic approaches confirmed by evidence-based medicine [2, 3]. There is a research discovering that ICH mainly occurs to people aged 40-70 [4]. Christensen et al. reported that ICH incidence is increasing year by year, which causes great psychological pressure and economic burden to the family and society due to the nonrenewability of brain neurons and the severe neurological dysfunction of ICH patients [5]. Although the regular treatment and comprehensive management can significantly reduce mortality and improve the outcome of ICH, they can also seriously damage the nervous system at the same time [6]. At present, the most critical predictors of ICH include its volume, the age of patients, the amount of blood in the brain, and the neurological function score. The most common manifestation of ICH is the neurological deterioration, which can lead to death [7]. Therefore, the study on ICH is of great importance.

Long noncoding RNA (lncRNA), a class of RNA molecules with a length of more than 200 nt transcribed by RNA Pol II from independent promoters, does not encode proteins but can be transcribed and has specific functions, which is cell-and tissue-specific, low in sequence conservation in general while relatively conserved in the secondary structures [8]. The specificity of lncRNAs is highly expressed in the central nervous system. Some scholars have found that 849 out of 1328 lncRNAs exist in specific cell types and subcellular structures in the neural region, and multiple studies show that ischemic stroke induces changes in the expression of a large number of lncRNAs [9], suggesting that lncRNA is related to the complex pathological process of ischemic stroke. In recent years, a number of studies have also reported the key regulatory role of lncRNA as markers in the treatment of brain injury diseases such as ICH [10–12]. As a “star molecule,” lncRNA H19 has been manifested that its downregulation can reduce brain edema and alleviate brain damage as well as neurological injury when ischemia occurs [13]. Chen et al. [14] showed for the first time that lncRNA H19 expression was upregulated in ICH cell model. And lncRNA H19 downregulation could promote the proliferation of brain microvascular endothelial cells and inhibit ferroptosis, thus achieving the effect of treating ICH. However, Chen et al. only investigated the functional mechanism of lncRNA H19 in ICH from *in vitro* cellular experiments, and we believe that the function of lncRNA H19 has not been fully elucidated. In consequence, the present study focuses on the vivo experimental to explore the regulatory effect of lncRNA H19 on ICH and analyzes its possible mechanism to provide a reference basis for finding new biomarkers to assess the severity of ICH from aspects like neurological function, inflammatory factors, and NF-*κ*B pathway.

## 2. Materials and Methods

### 2.1. Experimental Rats and Grouping

A total of 24 8-9-week-old male Sprague-Dawley rats weighing 250-300 g were randomly divided into four groups with 6 rats in each group: sham group (sham operation group, no intracranial injection of type IV collagenase), ICH group (intracerebral hemorrhage model group, intracranial injection of type IV collagenase), sh-NC group (2 h after ICH modeling, injection of negative shRNA at the same injection site), and sh-H19 group (2 h after ICH modeling, injection of H19 shRNA at the same injection site). Rats were euthanized at 48 h after surgery, whose brain tissue and peripheral blood were collected then. This study was approved by the Animal Ethics Committee of Guangdong Medical Laboratory Animal Center (C202109-28).

### 2.2. ICH Model

An ICH model of rats was modified according to the method of Rosenberg et al. [15]. The rats were anesthetized with intraperitoneal injection of 2% pentobarbital sodium (30 mg/kg). Type IV collagenase (0.2 U in *μ*l of sterile normal saline; Sigma-Aldrich, Germany) was slowly injected into the right caudate nucleus with a microinjector. After the injection, the needle was retained for 10 min and then slowly withdrawn, and the wound was cleaned, disinfected, and sutured. Throughout the whole modeling procedure, the anal temperature of the rats was maintained at 37°C-38°C. After the surgery, the rats were kept in a 25°C incubator.

### 2.3. Neurological Function Score of Rats

Neurological impairment in rats was evaluated by Rosenberg scoring standard [15]. 0 point: there were no signs of nerve injury; 1 point: the lateral forelimbs were flexed under the abdomen while the normal lateral forelimbs were extended to the ground when the rats were lifted; 2 points: in addition to the signs of 1 point, the resistance of pushing the paralyzed side of rats was significantly lower than that of pushing the contralateral side; 3 points: except for the above signs, the rats had the phenomenon of tail pursuit. 4 points: the activity of the rats was mainly rotated to the paralyzed side, and the active activity was obviously decreased. A score over 2 points indicated the success of model building.

### 2.4. Determination of Brain Water Content

The water content of the rat brain was determined on the third day after the establishment of an ICH model of rats [16]. After the rats were euthanized by 2% pentobarbital sodium (50 mg/kg), their heads were directly taken without perfusion and their brain tissues were dissected out. Next, the brain tissues were rapidly divided into three parts: the lesion and the contralateral side as well as the cerebellum, which were weighed on an electronic balance to obtain a wet weight to be recorded. Afterwards, the brain tissues were transferred to a 100°C oven and weighed again after 24 h to obtain a dry weight. The brain water content was calculated as follows: (wet weight − dry weight)/wet weight × 100%.

### 2.5. ELISA Detection

The serum was taken from rats in each group. Then, the contents of myelin basic protein (MBP), S-100B, and neuron-specific enolase (NSE) in the serum and the levels of inflammatory cytokines TNF-*α*, IL-6, and IL-1*β* in brain homogenate were detected according to the instructions of the ELISA kit (Nanjing Jiancheng Bioengineering Institute Co., Ltd.).

### 2.6. Determination of SOD, MDA, and ROS

The activity of SOD and the contents of MDA and ROS in the perihematoma tissues of rat brain in each group were determined by Superoxide Dismutase (SOD) assay kit, Malondialdehyde (MDA) assay kit, and Reactive oxygen species (ROS) assay kit (Nanjing Jiancheng Bioengineering Institute, China) according to the operating instructions.

### 2.7. Quantitative Real-Time Polymerase Chain Reaction (qRT-PCR)

Total RNA from brain tissue was extracted using the TRIzol kit (15596-018, Beijing Solarbio Science & Technology Co., Ltd., USA). RNA was then reverse transcribed into cDNA with SuperScript III Reverse Transcriptase (Invitrogen, USA) kit. Under the manufacturer's protocol, qRT-PCR assay was performed by the SYBR® Premix Ex TaqTM II kit (TaKaRa, Japan), with GAPDH as an internal control for lncRNA. The relative transcription level of the target gene was calculated using the 2^-△△CT^ method. Three replicate wells were set up for each sample, and each experiment was repeated three times. lncRNA H19 primer sequences were as follows: forward 5′-GATGACAGGTGTGGTCAACG-3′ and reverse 5′-CAGACATGAGCTGGGTAGCA-3′.

### 2.8. Western Blot

Total protein was extracted from the rat brain tissue, quantified by BCA, and separated by 10% SDS-PAGE electrophoresis. The proteins were subsequently transferred to PVDF membrane and blocked with blocking solution containing 5% nonfat dry milk for 1 h. The membranes were then incubated with the primary antibody NF-*κ*Bp65 (ab16502, Abcam, UK), IKK*β* (ab32041, Abcam, UK), and I*κ*B*α* (sc-1643, Santa Cruz Biotechnology, USA) overnight at 4°C. Then, the membranes were washed with TBST 3 times, and secondary antibody (1 : 2000, Abcam) marked by HRP was added to incubate at room temperature for 2 h. After TBST washed again, ECL luminescence agent (Sigma, USA) was evenly instilled and the gel imaging system was used for scanning analysis.

### 2.9. Statistical Analysis

Statistical analysis of the data in this study was performed by the SPSS 21.0 statistical software. Experimental data were expressed by mean ± standard deviation (SD), group comparison using one-way ANOVA as well as repetitive measurement analysis of variance, and pairwise comparison within one group using *t*-test. *p* < 0.05 was considered to have a statistical significance.

## 3. Results

### 3.1. High Expression of lncRNA H19 in Brain Tissue of ICH Rats

The results of qRT-PCR assay revealed (Figure 1) that compared with the sham group, the expression level of lncRNA H19 in the brain tissue of the ICH group was significantly increased; compared with the sh-NC group, the expression level of lncRNA H19 in the sh-H19 group was notably reduced. There was no significant difference between the ICH group and the sh-NC group (*p* > 0.05). The results confirmed that lncRNA H19 may be involved in the occurrence of ICH.

### 3.2. Inhibition of Nerve Injury in the Brain Tissue of ICH Rats by Interfering lncRNA H19

The effect of the expression of lncRNA H19 on brain tissue injury in ICH rats was further determined. The neurological assessment showed (Figure 2(a)) that the score of the sham group was 18, and the score of the ICH group was significantly lower compared with it (*p* < 0.05); the score of the sh-H19 group was higher compared with the sh-NC group (*p* < 0.05). Meanwhile, the water content in the perihematoma tissue of the ICH group was increased compared with the sham group; the water content in the sh-H19 group was greatly decreased compared with the sh-NC group (Figure 2(b)).

In addition, ELISA detection indicated (Figures 2(c)–2(e)) that compared with the sham group, the contents of MBP, S-100B, and NSE in the serum of rats in the ICH group were significantly enhanced; however, the contents of them in the sh-H19 group were lower than those in the sh-NC group. These results proved that interference with the expression of lncRNA H19 inhibited neural injury in the brain tissue of ICH rats.

### 3.3. Inhibition of the Expression of Inflammatory Factors in the Brain Tissue of ICH Rats by Interfering lncRNA H19

The results of ELISA assay manifested (Figures 3(a)–3(c)) that the levels of TNF-*α*, IL-6, and IL-1*β* in the perihematoma tissue of rats in the ICH group were remarkably increased when compared with those in the sham group; in comparison, the levels of TNF-*α*, IL-6, and IL-1*β* in the tissues after interference with lncRNA H19 were obviously decreased compared with those in the sh-NC group, which suggested that the low expression of lncRNA H19 inhibited the inflammatory injury in the brain tissue of ICH rats.

### 3.4. Inhibition of Oxidative Damage in the Brain Tissue of ICH Rats by Interfering lncRNA H19

Compared with the sham group, the levels of ROS and MDA were increased while SOD activity was decreased in the perihematoma tissue of rats in the ICH group; compared with the sh-NC group, the levels of ROS and MDA were higher while SOD activity was lower in the tissue of the sh-H19 group (Figures 4(a)–4(c)), which implied that the low expression of lncRNA H19 inhibited oxidative damage in the brain tissue of ICH rats.

### 3.5. Inhibition of the Activation of NF-*κ*B Signaling Pathway by Interfering lncRNA H19

It has been confirmed that NF-*κ*B signaling pathway plays an important role in secondary injury after cerebral hemorrhage [17]. Therefore, we further investigated the effect of lncRNA H19 expression on NF-*κ*B signaling pathway. Western blot (Figure 5) showed that the expression levels of NF-*κ*Bp65 and IKK*β* were increased, and the protein expression of I*κ*B*α* was decreased in the pericentral hematoma tissues of ICH rats compared with the sham group; by comparison, the expression levels of NF-*κ*Bp65 and IKK*β* were decreased and the protein expression of I*κ*B*α* was increased in the tissues of the sh-H19 group compared with the sh-NC group.

## 4. Discussion

ICH, being the most serious type of stroke, is the main cause of death and disability, and the research strategies on its targeted treatment are limited so far [2]. Niu et al. pointed out that alleviating brain injury and improving neuronal survival rate have been proposed as a key to the treatment of ICH [18], so lncRNA is regarded as a therapeutic target [19]. It was found that lncRNA H19 can play a specific function in brain development and diseases [13], but the study of lncRNA H19 regulating brain injury in ICH rats has not been reported. In this study, lncRNA H19 was highly expressed in the brain tissue of ICH rats. Therefore, we speculated that lncRNA H19 was involved in ICH occurrence.

The neurological function score is a common index for clinical evaluation of the therapeutic effect of ICH. There was a study that the behavioral changes of rats with ICH after successful modeling are consistent with their evolution of brain edema [20]. It was found in this study that the neurological function score of rats in the ICH group was significantly reduced, with the water content of tissues around the brain hematoma being increased. However, the brain function score was increased with the water content of tissues being reduced after interference with lncRNA H19 expression. S-100B protein, NSE (neuron-specific enolase), and MBP (myelin basic protein) have received much attention as neuron-specific serum markers and are considered to be high specific for assessing the damage of central nervous system and important for the evaluation of prognosis [21]. In the present study, the contents of MBP, S-100B, and NSE were obviously elevated in the serum of rats in the ICH group, while the contents of them were notably declined after interference with lncRNA H19 expression. As a result, it was hypothesized that lncRNA H19 might aggravate neurological impairment in the rat brain.

Inflammation plays an important role in hemorrhagic brain injury. Hence, the expression of inflammatory factors will be accompanied in the process of ICH, especially IL-1*β*, TNF-*α*, IL-8, and IL-6, which can change the permeability of blood-brain barrier [22]. In this study, the content of inflammatory factors (TNF-*α*, IL-6, and IL-1*β*) in perihematoma tissues of ICH rats was increased, while the content of them (TNF-*α*, IL-6, and IL-1*β*) in the sh-H19 group was decreased, which illustrated that silencing the expression of lncRNA H19 could inhibit the release of proinflammatory factors and thereby alleviate the secondary inflammatory response of ICH. Besides, ICH also affects oxidative stress response. Reactive oxygen species, superoxide dismutase, and malondialdehyde can not only reflect the important parameters of the body's antioxidant potential but also reflect the degree of tissue damage [23]. It was further discovered that silencing lncRNA H19 could significantly reduce the contents of MDA and ROS in brain tissue of ICH rats and enhance SOD activity.

In the central nervous system, NF-*κ*B signaling pathway mainly exists in neurons, glial cells, and vascular endothelial cells [24], which is composed of NF-*κ*B family, I*κ*B family, and IKK complex. IKK/NF-*κ*B signaling pathway is one of the most important inflammatory pathways found in current studies. In the middle cerebral artery occlusion (MCAO) animal model of cerebral ischemia, oxidative stress after cerebral ischemia induces a large number of IKK*α* to aggregate in the nucleus. IKK*α* and IKK*α*/*β* are, respectively, phosphorylated at 1 h and 24 h after operation, and I*κ*B is activated, so that NF-*κ*Bp65 subunit is dissociated into the nucleus and binds to the target gene to promote the expression of inflammatory factors [25]. A research has shown that the expression of IKK*β* protein began to increase half an hour after spinal cord injury. After inhibiting the phosphorylation of pI*κ*B*α* and the activity of IKK*β*, the activity of NF-*κ*B was also inhibited, thereby reducing the infiltration of inflammatory cells and reducing the apoptosis in spinal cord tissue [26]. In this study, it was found that after silencing lncRNA H19, the expression of NF-*κ*Bp65 and IKK*β* in the brain tissue of ICH rats was decreased, and the expression of I*κ*B*α* was increased, indicating that lncRNA H19 could lead to neurological damage, release inflammatory factors, exacerbate oxidative stress, and further aggravate the brain injury of ICH rats by activating the NF-*κ*B pathway. However, further studies are needed on the regulatory pathway through which lncRNA H19 activates the NF-*κ*B signaling pathway involved in mediating brain injury in rats.

## 5. Conclusion

In summary, knockdown of lncRNA H19 inhibited neurological impairment and brain edema and suppressed inflammatory response and oxidative stress, which in turn ameliorated brain injury in ICH rats. This was associated with inhibition of NF-*κ*B signaling pathway activity.

## Figures and Tables

**Figure 1:** lncRNA H19 was upregulated in brain tissue of ICH rats. The expression of lncRNA H19 in the perihematoma tissues of rats in each group was determined by qRT-PCR. *N* = 6 per group. ^∗∗∗^*p* < 0.001 vs. the sham group; ^##^*p* < 0.01 vs. the sh-NC group. ICH: intracerebral hemorrhage.

**Figure 2:** Inhibition of nerve injury in the brain tissue of ICH rats by interfering lncRNA H19. (a) Neurological deficit scores of rats in each group. (b) Determination of water content in perihematoma tissue of rats in each group. (c–e) ELISA determination of the levels of (c) S-100B, (d) neuron-specific enolase (NSE), and (e) myelin basic protein (MBP) in the serum of rats in each group. *N* = 6 per group. ^∗∗^*p* < 0.01 and ^∗∗∗^*p* < 0.001 vs. the sham group; ^#^*p* < 0.05 and ^##^*p* < 0.01 vs. the sh-NC group. ICH: intracerebral hemorrhage.

**Figure 3:** Inhibition of the expression of inflammatory factors in the brain tissue of ICH rats by interfering lncRNA H19. The contents of (a) TNF-*α*, (b) IL-6, and (c) IL-1*β* in the perihematoma tissue of rats in each group were detected by ELISA. *N* = 6 per group. ^∗∗^*p* < 0.01 and ^∗∗∗^*p* < 0.001 vs. the sham group; ^#^*p* < 0.05 and ^##^*p* < 0.01 vs. the sh-NC group. ICH: intracerebral hemorrhage.

**Figure 4:** Inhibition of oxidative damage in the brain tissue of ICH rats by interfering lncRNA H19. The levels of (a) malondialdehyde (MDA), (b) reactive oxygen species (ROS), and (c) superoxide dismutase (SOD) activity in perihematoma tissue of rats in each group were determined. *N* = 6 per group. ^∗∗∗^*p* < 0.001 vs. the sham group; ^##^*p* < 0.01 vs. the sh-NC group. ICH: intracerebral hemorrhage.

**Figure 5:** Inhibition of the activation of NF-*κ*B signaling pathway by interfering lncRNA H19. The expressions of NF-*κ*Bp65, IKK*β*, and I*κ*B*α* in the perihematoma tissues of rats in each group were detected by Western blot. The experiment was repeated three times. ^∗∗∗^*p* < 0.001 vs. the sham group; ^##^*p* < 0.01 vs. the sh-NC group. ICH: intracerebral hemorrhage.

## Data Availability

The data used to support the findings of this study are available from the corresponding author upon request.
